The article "A Novel Method of Clinical Nursing under the Medical Internet of Things Technology" was retracted in 2023. Reasons: signs of a paper mill; suspected computer-generated content; unreliable results or conclusions; lack of ethics approval or compliance.

# A Novel Method of Clinical Nursing under the Medical Internet of Things Technology

**DOI:** 10.1155/2021/2234457

**Published:** 2021-11-09

**Authors:** Tingting Ou, Xuehua Cai, Meichun Wang, Feirong Guo, Biyu Wu

**Affiliations:** ^1^Vascular Channel Nursing Specialist Clinic, Quanzhou First Hospital, Quanzhou 362000, China; ^2^Outpatient Department, Quanzhou First Hospital, Quanzhou 362000, China; ^3^Nursing Department, Quanzhou First Hospital, Quanzhou 362000, China

## Abstract

Internet of things technology began to spread to all industries of our lives; the application of medical internet of things in many hospitals highlighted its advantages and brought a lot of convenience to patients and medical staff. With the continuous progress of China's medical reform and the continuous improvement of patients' requirements for medical service quality, this paper discusses the application of medical internet of things in clinical nursing in ward, and the basic information collection, infusion, and mobile nursing were discussed and studied. Through the parallel control study of the laboratory itself, this paper evaluates whether the two different clinical measurement methods of medical internet of things technology and traditional technology are consistent in body temperature, pulse, respiration, and blood oxygen saturation. At the same time, it also deeply studies the value and advantages of internet of things technology in the application of other monitoring indicators in clinical nursing and analyses the problems in its application. The experimental data show that the two measurement methods with different principles can be completely replaced in clinical application, and the time efficiency of the new clinical nursing method under the medical internet of things technology in mapping body temperature, pulse, and respiration has been improved by 76.20% and 72.02%, respectively, surpassing the traditional information technology and realizing the intelligent, automatic, and standardized data acquisition method. It ensures the authenticity of data and the real-time of information flow and meets the needs of resource sharing and medical regional interconnection.

## 1. Introduction

Due to the complexity and breadth of clinical nursing work, the collection of transactional nursing information occupies a lot of manpower, material resources, and time; the computer processing process of nursing information has high requirements for information processing methods and technologies. Nursing information has different attributes and different processing methods. Highly subjective information must be collected and recorded on site by nurses with professional knowledge and stored on paper carriers or mobile devices [1]. The objective information is collected one by one by the nursing staff carrying measuring instruments to the patient's bedside and then recorded manually. After completing the information collection, it is returned to the nursing station for classification and processing, and part of it is input into the computer nursing information database for storage, analysis, and re-extraction so as to realize nursing information management [2]. The other part is kept in the form of paper materials, and the nursing management personnel carry out quality control afterwards. On the one hand, nurses must participate in many links of data processing in the whole process; on the other hand, they must complete complicated manual operation and nursing tasks such as treatment, observation, and feedback at the same time. Its high labour intensity, low efficiency, high error rate, and low value embodiment making nurses in a high-tension working state for a long time, resulting in high work pressure and serious job burnout [3]. From the perspective of patients, clinical diagnosis, and treatment, nursing data from collection, analysis, cleaning, and storage to the final service application have obvious periodicity and lag, which cannot provide necessary dynamic data for clinical nursing diagnosis and treatment and affect the accuracy of clinical nursing diagnosis and treatment decision-making and effect [4]. From the perspective of information equipment, restricted by the advanced degree and the relatively fixed mobile range of equipment, the efficiency of medical treatment will be affected to varying degrees in the process of information processing, which will complicate the workflow, and there is a situation that the information process and the medical care process are seemingly inseparable [5]. The above phenomena truly reflect the current situation and level of clinical nursing information management and are also the doubts and difficulties that must be faced and solved in the in-depth application of the nursing information management system [6].

The article "A Novel Method of Clinical Nursing under the Medical Internet of Things Technology" was retracted in 2023. Reasons: signs of a paper mill; suspected computer-generated content; unreliable results or conclusions; lack of ethics approval or compliance.

The organic integration of internet of things and nursing activities is one of the important characteristics of nursing development in the 21st century. The advantage of the application of the internet of things in clinical nursing lies in that the information receiver with sensors replaces people to “perceive” the information of human body, facilities, and environment and is not limited by time and space [7]. It can automatically collect, transmit, and process real-time information comprehensively, efficiently, dynamically, continuously, and conveniently and synchronously realize the functions of real-time analysis and decision support [8]. This has become an opportunity for the innovative development of clinical nursing. Due to the characteristics of thorough perception, comprehensive interconnection, and intelligent insight of the internet of things, it can realize the tracking and supervision of the whole process of medical and nursing affairs and clinical nursing business, expand the coverage of clinical nursing business, management, and service, and comprehensively systematize intelligent medical treatment, precision nursing, and quality service [9]. The goal of clinical nursing work is made more efficient and convenient; complete, true, and reliable judicial evidence is provided for handling medical disputes or accidents; it also provides an objective basis for scientific evaluation to improve nursing value and highlight nursing quality level and management benefit [10]. Based on this research background, the innovative development and value of internet of things technology to clinical nursing are further thought. How to achieve the timely, accurate, efficient, and standardized collection of clinical nursing information, particularly after integration with the nursing information management system, and the degree of high integration and sharing, directly affect the level of nursing quality [11].

This paper aims at the current situation that the traditional methods have high labor intensity, low efficiency, high error rate, and low value embodiment, which makes the nurses in a high-tension working state for a long time, thus affecting the accuracy of clinical nursing diagnosis and treatment decision-making and effect, discusses the application of medical internet of things in clinical nursing in ward, and discusses and studies the basic information collection, infusion, and mobile nursing. Through the parallel control study of the laboratory itself, this paper evaluates whether the two different clinical measurement methods of medical internet of things technology and traditional technology are consistent in body temperature, pulse, respiration, and blood oxygen saturation. At the same time, it also deeply studies the value and advantages of internet of things technology in the application of other monitoring indicators in clinical nursing and analyses the problems in its application. The experimental data show that the two measurement methods with different principles can be completely replaced in clinical application, and the mapping efficiency of the new clinical nursing method under the medical internet of things technology exceeds the traditional information technology, realizes the intelligent automation and standardized data acquisition method, and ensures the authenticity of data and the real-time of information flow; it meets the needs of resource sharing and medical regional interconnection.

The article "A Novel Method of Clinical Nursing under the Medical Internet of Things Technology" was retracted in 2023. Reasons: signs of a paper mill; suspected computer-generated content; unreliable results or conclusions; lack of ethics approval or compliance.

The chapters of this paper are arranged as follows.  Section 1 summarizes the research background and significance of this paper.  Section 2 introduces the internet of things-related technologies.  Section 3 analyses the implementation ways of new methods for the application of medical internet of things technology in clinical nursing.  Section 4 carries out experimental analysis, and Section 5 summarizes the full text.

## 2. Relevant Technologies of Internet of Things

### 2.1. Overall Structure

With the development of technology and application, the connotation and extension of the concept of internet of things are also expanding. Its overall framework includes the following five parts, namely, community architecture, technological know-how system, preferred system, associated enterprise device, and useful resource system. The terminal sensing layer consists of sensing terminal devices, such as RF readers, electronic tags, cameras global positioning system, and various sensors, and other sensing terminals collect data information [12]. The sensing terminal is equivalent to the peripheral nerve in the human structure, such as the human facial features. It is the terminal source for the internet of things to identify objects and collect information [13]. The community transmission processing layer, additionally acknowledged as the community layer, transmits the records and statistics amassed by way of the grasp layer to the vacation spot safely, rapidly, and reliably through the internet, conversation community, and community cloud platform. The network transport layer is equivalent to the command centre in the human structure, such as the central nerve and brain, which is responsible for the transmission and processing of information collected by the sensing terminal. Intelligent application layer: it is a bridge connecting the internet of things and users [14]. Users can be people, other systems, and organizations. It is used to analyse and process the information obtained by the sensing terminal and realize the intelligent application of the internet of things in combination with the needs of the industry, as shown in Figure 1.

### 2.2. Significance of Internet of Things in Clinical Nursing

The application of internet of things technology in the hospital nursing information system is of great significance and value. First, internet of things technology can quickly evaluate patients and accurately grade patients. Based on the internet of things technology, the preinspection system is set at the same time. The preinspection system can effectively, quickly, and accurately obtain patient information and conduct triage according to the severity of patients' diseases [15]. In addition, the patient information can be transmitted to doctors in real-time through the internet of things system, which can improve the efficiency of patients' treatment. In addition, the application of internet of things technology in the nursing information system can timely transmit patient information to rescue nurses; nurses can get information in time and implement rescue in time. Second, internet of things technology is conducive to improve nurses' work efficiency [16]. At the same time, the application of internet of things in the nursing information system can significantly reduce the incidence of errors. On the basis of internet of things technology, smart wristbands can be used to wear smart wristbands for newly admitted patients without bedside cards. Patients can be identified through wristbands, which not only facilitate nurses but also save time and improve work efficiency. By using smart watches for patients in the hospital, it can ensure that nurses work orderly and can be busy without disorder [17]. In addition, shrewd identification via the web of matters can radically decrease medicinal drug errors, keep away from patients' blunders in executing clinical orders, and extensively enhance the pleasant of work [18]. Third, the internet of things provides transparent data through the communication layer, obtains the physiological information of patients through the perception layer, and can reflect the information to nurses through the network layer. Nurses do not need to use traditional instruments to monitor the vital signs of patients and do not need to arrive at the patient's bed every hour or 30 minutes to collect information. Nurses solely accumulate the patient's existence signs and symptoms and situation modifications via the screen and wise show screen and transmit the patient's atypical facts to doctors, so as to facilitate analysis and treatment, improve the patient's cure probability, and effectively protect the patient's life and health [19].

The article "A Novel Method of Clinical Nursing under the Medical Internet of Things Technology" was retracted in 2023. Reasons: signs of a paper mill; suspected computer-generated content; unreliable results or conclusions; lack of ethics approval or compliance.

### 2.3. Specific Application of Medical Internet of Things

Combined with the previous design, the internet of things network based on Wi-Fi and RFID technology is designed to realize specific applications. In this project, the medical internet of things is selected as the final technical landing point. The application environment and conditions of medical internet of things are as follows: Wi-Fi signal coverage has been realized in the ward environment, and the nurse workstation has network access to the hospital LAN. The hospital has its own database system; according to the environment and requirements, the overall structure of the designed medical internet of things network is shown in Figure 2.

In this system, the sphygmomanometer, as a sensor node, has RFID read-write function and Wi-Fi communication function. In use, the sphygmomanometer first collects the patient's personal information in the label, then measures the patient's blood pressure data by the Coriolis auscultation method, and then connects the Wi-Fi network through the wireless access point to bind the patient information and blood pressure data and send them to the nurse station PC; the PC runs the application software to further save the data to the hospital database system [20]. Through the analysis of the system, the main contents of the work are in two aspects: the design of sphygmomanometer terminal and the preparation of nurse workstation application software. The application software has been written by other students, so the focus of the work is mainly on the design of sphygmomanometer terminal.

## 3. A New Method for the Application of Medical Internet of Things Technology in Clinical Nursing

### 3.1. System Design

According to the needs of clinical nursing and the application environment of the system, the following problems must be solved in the system design. (1) *Portable Device.* The sensor is concentrated in a portable device with high reliability, which meets the requirements of small volume and convenient use and has the performance of high measurement accuracy. (2) *Low-Power Consumption*. Due to the frequent use of sensing terminal equipment, but the amount of data collected is small and no high transmission rate is required, low-power consumption can ensure a long service time of the equipment without frequent charging [21]. (3) *Automatic Networking*. Each ward has at least 40 beds, so at least 40 sets of sensing terminal equipment shall be allocated. These 40 sets of equipment shall automatically form a network and send vital signs parameters to the server through wireless mode. (4) *Expansibility*. The environment of the ward is complex, there are many interference factors, and the environment and area of each ward are different. Therefore, it is necessary to ensure that the sensing terminal equipment can be used in different environments and has high expansion performance. Through the investigation of existing communication technology in the early stage and combined with the characteristics of the current hospital information system, the system structure developed is shown in Figure 3. The ward intelligent nursing system mainly includes: electronic thermometer with wireless communication function and two-parameter measuring instrument of pulse and blood pressure. Through the physiological signal acquisition equipment in the hands of patients and the wireless gateway deployed in the ward corridor, the physiological parameter information is transmitted to the hospital information system to realize the intelligent acquisition of physiological parameters in the ward [22].

The article "A Novel Method of Clinical Nursing under the Medical Internet of Things Technology" was retracted in 2023. Reasons: signs of a paper mill; suspected computer-generated content; unreliable results or conclusions; lack of ethics approval or compliance.

In terms of technical implementation, the research and development of nRF905 low-power RF communication module with 433 MHz communication frequency band are focused. Combined with low-power MCU and physiological signal sensing equipment, it collects, analyses, and processes three key parameters that must be measured every day in the general ward: blood pressure, body temperature, and pulse. Accordingly, wireless electronic thermometer and wireless blood pressure pulse meter are developed in the sensing layer. The network realizes the conversion of RF communication into Wi-Fi communication and enhances the functions of temporary storage and automatic networking. In the application layer, the key physiological signal nursing system based on PDA and the real-time acquisition and control system based on PC are made.

### 3.2. Design of Sensor Layer

The body temperature sensor is mainly composed of temperature measurement circuit, main control chip, wireless transmission module, and power management module. The temperature measurement circuit is mainly composed of chip and thermistor. The main control chip of TI company and the wireless transmission module is nRF905 module [23, 24]. The temperature measurement chip converts the temperature into an electrical signal. The main control chip reads the electrical signal by interrupting and calculates the pulse data of the OEB pin of chip to read the temperature data. The main control chip judges whether the temperature is the maximum temperature by interrupt counting and saves it when it is the maximum temperature. When the main control chip gets the stable maximum temperature, it starts to configure the wireless transmission module to reduce the power consumption of the system and prolong the service time of the battery. When designing the temperature sensor, the following points must be considered: (1) it must meet the requirements of medical temperature measurement, and the measurement error is less than 0.1°C; (2) it has simple operation, anyone can use the thermometer quickly; (3) the shell is sealed, and the surface is smooth and has the functions of bacteriostasis and antidisinfection; (4) data transmission and control do not need manual participation and interference; (5) the measurement error compensation function is designed to solve the problem of temperature drift caused by thermistor aging; and (6) it has low-power consumption and extended battery life [25].

The article "A Novel Method of Clinical Nursing under the Medical Internet of Things Technology" was retracted in 2023. Reasons: signs of a paper mill; suspected computer-generated content; unreliable results or conclusions; lack of ethics approval or compliance.

The sphygmomanometer adopts a high-performance sound pressure sensor to judge the blood pressure value by extracting the Coriolis sound signal of auscultation. This method can eliminate the individual difference of the oscillography electronic sphygmomanometer and improve the accuracy of blood pressure measurement. In the design process, the Coriolis tone delay time technology is developed to further accurately determine the systolic and diastolic blood pressure and ensure the accuracy of individual measurement. High precision pressure sensor and customized Coriolis sound sensor are used to extract blood pressure related signals, and the overall performance of the system is improved through linear deflation and automatic pressure zeroing. The appearance of the mercury manometer is simulated by liquid crystal, with high scale resolution [26, 27]. It can accurately display the cuff pressure and observe the pulsation signal of the cuff. The functions of automatic data storage, playback, and analysis are realized. It has RF wireless transmission interface to realize the interconnection of Internet of things. The principle of pulse and sphygmomanometer is shown in Figure 4.

### 3.3. Design of Application Layer Service Software

The main functions of application layer service software are maintenance, display, collection, writing, viewing, and alarm of life parameter information. The maintenance function is mainly used for database maintenance, including adding, deleting, and updating records. The man-machine interface of the system is written based on C++ language, and the development tool is MFC application program based on VC++ 6.0 dialog box class [28]. The basic process is to discharge the basic information of patients in the ward from the hospital HIS, including patients' ID numbers, bed numbers, room numbers, diagnostic information, and attending doctors; nurses and doctors can intuitively see the patient's information [29]. When the life parameters are transmitted to the PC or server, they can be displayed to the interface in real-time. After receiving, the doctor or nurse can click the save button to save the parameter data to the server. The received data are displayed in the column corresponding to the patient [30]. When saving, it is also saved according to the patient's information. There will be no dislocation between the patient and vital signs parameters. The man-machine interface can also modify the number of the sensing terminal equipment. When the patient's equipment is damaged, the equipment can be replaced for the patient in time [31, 32]. The database adopts the link mode to connect the application software to the Oracle database in the background of the hospital and then executes the corresponding database programming statements to complete the reading and saving of the database and realize the operation of the fields in the corresponding table.

The article "A Novel Method of Clinical Nursing under the Medical Internet of Things Technology" was retracted in 2023. Reasons: signs of a paper mill; suspected computer-generated content; unreliable results or conclusions; lack of ethics approval or compliance.

## 4. Experiment and Analysis

Under the condition of overcoming individual differences, the experimental research design scheme of self parallel control is adopted. With the help of traditional measurement tools and medical internet of things, the control group and experimental group are set. The same person collects four vital sign parameters, body temperature, pulse, respiration, and blood oxygen saturation at 7 different time points in a day. This experiment is aimed at healthy groups to verify the feasibility and accuracy of the new technology in clinical nursing application. For the above data management work, the personnel in charge of nursing division or above shall be invited to guide and participate in data quality control, supervision, and management. Because the data collected by the two methods of comparison have the characteristics of point and surface differences, the latter is processed by the mean method and then compared. SPSS 22.0 statistical software was used to analyse the continuous repeated measurement data collected in the experiment by analysis of variance, paired *t* test, correlation coefficient, and Bland Altman method.

After the experiment, the data stored in the medical IoT system were transferred, and the tables were counted after counting. Finally, the recorder shall fill in the comparison form uniformly and the supervisor shall check it. The experiment is started after completing the pre-experiment. First, the data are entered into excel by the double entry method and then imported into SPSS 22.0 software for statistical analysis and description. The analysis of variance is used to understand the difference between the two groups of data, and the degree of difference is statistically described by paired *t* test, and then the correlation test is carried out for the two groups of data samples to understand the degree of correlation and bias. The above analysis of variance shows that the data of two different principal measurement methods of *R* are completely consistent, and there is no statistical difference, while the data of temperature, pulse, respiration, and blood oxygen saturation are not completely consistent, and there are statistical differences. With the help of the plot's submenu, the mean change trend diagram of the indicators measured repeatedly for 7 times is made, and the linear correlation regression equation of temperature and pulse is calculated, as shown in Figure 5. The temperature and pulse data meet the linear correlation analysis conditions, there is no obvious abnormal value, and the correlation coefficient is statistically significant.

The article "A Novel Method of Clinical Nursing under the Medical Internet of Things Technology" was retracted in 2023. Reasons: signs of a paper mill; suspected computer-generated content; unreliable results or conclusions; lack of ethics approval or compliance.

*F* = 8.504, *P*=0.005 ≤ 0.005, there is no linear correlation, and the control data of the two groups are different. The blood oxygen saturation results of control group (ECG) and experimental group (medical internet of things) were 98.00 ± 0.52 and 98.63 ± 0.81. Due to the difference in precision between the two different methods, it is necessary to further analyse the data in combination with clinical application standards. Therefore, the Bland Altman analysis method is used to evaluate the consistency of the two different measurement methods, and the calculated results are shown in Figure 6.

The difference between the measurement results of the two different methods is described by paired *t* test, as shown in Figure 7. Although the results of the two measurement methods are not completely consistent, there is always a certain deviation difference that the consistency of medical internet of things values is often greater than that of the control group, and there is a linear correlation between the two groups of data, indicating that the linear relationship between the two-control data is close and consistent. Through the analysis of the above statistical methods, the measurement results of the two measurement methods in the control group and the experimental group (medical internet of things) on the four parameters of temperature, pulse, respiration, and blood oxygen saturation are consistent; that is, the two methods can replace each other.

Through data analysis and clinical consistency evaluation, it is concluded that these two different measurement methods can completely replace each other in the accuracy of temperature, pulse, respiration, and blood oxygen saturation measurement, and the accuracy and sensitivity of medical internet of things are higher. The medical internet of things is fully used, highly operable, highly accepted by patients, and has strong clinical practicability and popularization. Under the internet of things technology, the integration of temperature, pulse, respiration surveying, and mapping in the three nursing test sheets has improved the time efficiency by 76.20% and 72.02%, respectively, compared with the traditional surveying and mapping methods 1 and 2. Time comparison of different surveying and mapping methods is shown in Figure 8.

Intelligent automation and standard dynamic data collection are realized in information collection, highlighting the advantages of standard collection, unified access, and transmission, data sharing, and unified service. It shortens the operation time of nurses' manual measurement of temperature, pulse, and respiration, reduces the error rate of data input system, and reduces the process links of vital signs measurement and drawing. In terms of monitoring human physiological parameters, it is more widely used and more powerful, convenient, and practical than the current ECG monitor. For example, the increased fall index, sleep index, and other more than a dozen indicators, including the noninvasive blood glucose and blood pressure monitoring channel to be opened soon, to comprehensively monitor the health status of patients, undoubtedly extend the nurse workstation to the patients and directly point the nursing safety management and nursing quality monitoring to the target of real-time dynamic management. It laid a solid foundation for realizing nursing scientific management and intelligent decision-making.

The article "A Novel Method of Clinical Nursing under the Medical Internet of Things Technology" was retracted in 2023. Reasons: signs of a paper mill; suspected computer-generated content; unreliable results or conclusions; lack of ethics approval or compliance.

The medical internet of things system in this test is seamlessly connected with NIS. Taking only one routine nursing work “mapping temperature, pulse, and respiration” as an example, the mapping efficiency of internet of things is about 76.2% and 72.02% higher than that of traditional methods (manual and semiautomatic). This result shows that the application of the new technology directly reduces the indirect nursing time. While improving the work efficiency and reducing the labour intensity, it also correspondingly reduces the office consumables. Especially, when a large number of patients are treated in the ward and temperature, pulse, and respiration surveyed, nurses will have a deeper experience in artificial intelligence mapping, which provides technical support for the transformation of the nursing workflow of collecting vital signs. In addition, compared with the traditional working mode, it highlights its strong artificial intelligence characteristics in the standardization, authenticity, correctness, timeliness, and sharing of data collection, which lays a solid foundation and rich resources for enriching the clinical nursing database system, and provides a scientific and safe guarantee for patient condition monitoring management, safety management, and high-quality service.

## 5. Conclusion

The use of medical internet of things in the ward can greatly improve the work efficiency of medical staff and reduce work errors. At the same time, it can also make the doctor-patient relationship more harmonious and improve the patient's nursing satisfaction. Medical internet of things can concentrate all information on the same platform so that resources can be used effectively; this paper designs and implements a new clinical nursing method based on medical internet of things. Based on the design principle of improving the automatic management level of hospital ward, reducing the work intensity of medical staff, reducing cost investment, and reducing patient bed accompanying, communication technology, photoelectric detection technology, microcomputer technology, computer network technology, and relational database technology are successfully applied to the ward intelligent monitoring system based on internet of things. The use of the system provides convenience for nurses' nursing work, provides a reliable safety guarantee for patients' daily treatment, and has high application value. The trial in several clinical wards shows that the system has high accuracy, stability, and consistency in the measurement of blood pressure, pulse, and body temperature. At the same time, both the sensor end and the application end can output reliable alarm signals when the data are abnormal or reach the warning value. Finally, the system is divided into multiple functional modules in a reasonable way, which can be customized and tailored to meet the application of different levels of hospitals or wards.

The article "A Novel Method of Clinical Nursing under the Medical Internet of Things Technology" was retracted in 2023. Reasons: signs of a paper mill; suspected computer-generated content; unreliable results or conclusions; lack of ethics approval or compliance.

## Figures and Tables

**Figure 1:** Architecture of internet of things.

**Figure 2:** Frame diagram of mobile nursing structure.

**Figure 3:** Intelligent monitoring system for ward.

**Figure 4:** Realize the medical internet of things interconnection of clinical nursing.

**Figure 5:** Correlation analysis of body temperature, pulse, respiration and blood oxygen saturation: (a) measured value of temperature; (b) measured value of pulse; (c) respiratory measurements; (d) monitoring value of blood oxygen saturation.

**Figure 6:** Comparison table of consistency evaluation: (a) evaluation of consistency; (b) comparison of limit value data.

**Figure 7:** Comparison of measurement results by different methods: (a) comparison of temperature; (b) comparison of pulse; (c) comparison of respiration; (d) comparison of blood oxygen saturation.

**Figure 8:** Time comparison of different surveying and mapping methods.

## Data Availability

The data used to support the findings of this study are included within the article.
